This article has been retracted.

# Tanshinone IIA May Inhibit Gastric Cancer via Affecting the Intestinal Microbiome

**DOI:** 10.1155/2022/6960304

**Published:** 2022-09-26

**Authors:** Fenggang Lu, Yi Zhang, Pinghui Song, Yu Xu, Zhongkun Wu, Qinyu Wang, Naiying Shen

**Affiliations:** Department of General Surgery, Shaanxi Health Care Group 215 Hospital, Shaanxi 712000, China

## Abstract

**Background:**

Gastric cancer (GC) belongs to a type of the most deadly cancer in the world, and the incidence rate of GC will increase in the coming decades. Tanshinone IIA (Tan IIA) is an active component that separated from Danshen. Tan IIA may also exert its therapeutic effects in disease with intestinal dysbacteriosis, at least partially, via regulating the intestinal microbiome. Nevertheless, it is obscure whether Tanshinone IIA affects the intestinal dysbacteriosis and plays antitumor roles. This research was designed to explore Tanshinone IIA potential on the intestinal dysbacteriosis of GC xenograft mice.

**Methods:**

Mouse xenograft GC tumor models were built and treated by Tan IIA. The tumor growth as well as microbiome in the intestinal were compared. Western blot was used to detect the phosphorylation of the NF-*κ*B and expressions of the downstream cytokines IL-6 and IL-1*β*.

**Results:**

Microbiome in the intestinal was changed in xenograft tumor mice in comparison with the control mice. What is more, Tan IIA could influence the microbiome in the intestinal of the tumor mice. Tan IIA hinders the growth of xenograft tumor and change the microbiome in the intestinal, but intestinal dysbacteriosis condition partially blocked Tan IIA-stimulated antitumor effects. In addition, intestinal dysbacteriosis abrogated Tan IIA-stimulated decrease in the NF-*κ*B signaling in xenograft tumor mice.

**Conclusions:**

Tanshinone IIA may inhibit GC tumor growth via affecting the intestinal microbiome through regulating the NF-*κ*B signaling.

## 1. Background

Gastric cancer (GC) belongs to a type of the most deadly cancer in the world, and the incidence rate of GC will increase in the coming decades [1, 2]. In spite of the recent advances in therapy, the long-time overall survival rate of GC is inferior to 10% [3, 4]. As a consequence, studying more methods for GC diagnosis and therapy is necessary.

Previous studies have proposed the possible role of gut microbiome in cancers [5, 6]. Intestinal dysbacteriosis, which is abnormal changes in the gut microbiota, may induce abnormal immune reaction in the gastric tissues, triggering the chronic inflammation and epithelial-mesenchymal transition (EMT) of the epithelial cells, ultimately stimulating tumor development [7]. Therefore, to alleviate the intestinal dysbacteriosis condition may be another way to treat various types of cancers.

Tanshinone IIA (Tan IIA) was an active component that separated from Danshen (a traditional medication) [8, 9]. Tan IIA has antiapoptotic, antioxidant, and anticoagulant along with other effects and has been extensively utilized in treating cardiovascular as well as cerebrovascular diseases. Recently, the antitumor potentials of Tan IIA have been discussed in many previous studies, including cancers [10]. Interestingly, a previous studied showed that the major bioactive parts of Danshen are tanshinones, which can exert medical effect in the rat chronic renal failure model by modulating the intestinal microbiome along with alleviating the intestinal dysbacteriosis [11]; moreover, tanshinol borneol ester, which is a bioactive component isolated from Danshen, can reverse the intestinal dysbacteriosis condition of high-fat diet-induced mouse obesity model [12]; furthermore, Danshen has been reported to restore the balance of intestinal microbiome and reduce the translocation of the microbiome in rat hepatic ischemia/reperfusion injury models [13].

The transcriptional factor nuclear factor-*κ*B (NF-*κ*B) family regulates a huge number of genes implicated in different cellular processes, such as cell proliferation, differentiation, and innate and adaptive immune responses. The NF-*κ*B family consists of 5 members, p50, p52, p65, RelB, and c-Rel, which interact to form homopolymers or heterodimers [14]. Activation of the NF-*κ*B signaling pathway contributes to the progression of several cancers, GC included [15]. Moreover, the NF-*κ*B signaling pathway plays a key role in the host response to microbial infection by coordinating innate and adaptive immune functions [16]. Since Tan IIA is an important bioactive component of the Danshen, according to the mentioned previous reports, we speculated that Tan IIA may also exert its therapeutic effects in a disease with intestinal dysbacteriosis, at least partially, via regulating the intestinal microbiome. Nevertheless, it is obscure whether Tanshinone IIA affects the intestinal dysbacteriosis and plays antitumor roles. Herein, we explored Tanshinone IIA role on the intestinal dysbacteriosis of GC xenograft mice and the underlying mechanism. Our work may offer a new mechanism along with an alternative treatment strategy for GC patients.

## 2. Methods

### 2.1. Cell Cultivation

Procell (Wuhan, China) supplied human gastric cell line HT29 (Cat. No. TCHu103), which were hatched in McCoy's 5A medium with 10% FBS at 37°C with 5% CO_2_.

### 2.2. Xenograft Tumor Models of HT29 Cells and Intestinal Dysbiosis Mouse Model

40 male mice (4-6 weeks old) from Animal Center of Nanjing Medical University (Nanjing, China) were spanided into 4 groups (*n* = 10 every group) in random (control group, Tan IIA high group, Tan IIA+dysbacteriosis group, and dysbacteriosis group). All procedures were conducted following the Guidelines for the Care and Use of Laboratory Animals with the approval of the Ethics Committee of the Shaanxi Health Care Group 215 Hospital. The mice were placed in a specific pathogen-free (SPF) condition, supplying water and food. For the xenograft tumor models, HT29 cells (2 × 10^6^ cells) with different treatments were subcutaneously injected into the mice. For Tan IIA treatment, low and high doses of Tan IIA were 10 mg/kg and 30 mg/kg, respectively. 21 days later, the mice were treated with isoflurane for anesthetizing and placed in a room with CO_2_ (flow rate < 30% volume/min) for 7 minutes for sacrifice. After excising the tumor tissues, the tumor was measured.

An intestinal dysbiosis mouse model has been built as previously documented [17]. Mice have been orally injected by ampicillin (1 g/l), vancomycin (0.5 g/l), neomycin (1 g/l), and metronidazole (1 g/l) to create intestinal dysbiosis condition.

### 2.3. Western Blotting

Total proteins were extracted and then isolated by a 10% SDS–PAGE. After shifting to PVDF membranes along with sealing in TBST solution including 5% skimmed milk, the membranes were hatched with primary antibodies including p-NF-*κ*B (Abcam, ab239882, 1/1000) and *β*-actin (Abcam, ab8226, 1 *μ*g/ml) and then hatched with HRP-conjugated secondary antibodies (Abcam, ab239882, 1/2000). Protein bands were examined via enhanced chemiluminescence detection system (Millipore, USA). Images are revealed as representatives of three independent assays.

### 2.4. ELISA Assay

The levels of interlukin-6 and interlukin-1*β* were measured by ELISA methods (Beyotime, Shanghai, China).

### 2.5. Statistical Analysis

All assays were implemented in triplicate. Data were indicated as mean ± SD and programed via SPSS 19.0 software. Comparison was assessed using unpaired Student's *t*-test. *p* value below 0.05 was meaningful.

## 3. Results

### 3.1. Changes of the Microbiome in the Intestinal of the Tumor Mice in Xenograft Tumor

First, we established the xenograft tumor mouse models, and the microbiome in the intestinal of the tumor mice and normal mice were compared. As illustrated in Table 1, the relative abundance of *Lactobacillus* as well as *Bacteroides* decreased (*p* < 0.01) and *Escherichia* as well as *Candidatus* markedly increased (*p* < 0.001) in tumor mice.

### 3.2. Tan IIA Hinders the Growth of Xenograft Tumor and Change the Microbiome in the Intestinal

Furthermore, to verify whether Tan IIA could repress the growth of xenograft tumor via modulating the microbiome in the intestinal, we treated Tan IIA into the xenograft tumor mice. As unveiled in Figure 1, the tumor size and weight were markedly decreased in the Tan IIA low and Tan IIA high groups relative to the control group (*p* < 0.05 and *p* < 0.01). At the same time, the tumor volume was gradually reduced at 14 and 21 days (*p* < 0.05 and *p* < 0.01). Moreover, Tan IIA elevated the abundance of *Lactobacillus* as well as *Bacteroides* and declined the abundance of *Escherichia* as well as *Candidatus* in a dose-dependent way (Table 2, *p* < 0.05 and *p* < 0.01).

### 3.3. Intestinal Dysbacteriosis Condition Partially Blocked Tan IIA-Stimulated Antitumor Effects

Next, an intestinal dysbiosis model was established by a large dose of antibiotics as previously described, and as Figure 2 showed, Tan IIA decreased the tumor growth; meanwhile, intestinal dysbiosis condition could partially block Tan IIA caused inhibition on the tumor growth in xenograft tumor mice (*p* < 0.05 and *p* < 0.01).

### 3.4. Intestinal Dysbacteriosis Abrogated Tan IIA-Stimulated Decrease in the NF-*κ*B Signaling in Xenograft Tumor Mice

Finally, to elucidate the possible mechanism of Tan IIA-induced antitumor effects via regulating the microbiome in the intestinal, the phosphorylation of the NF-*κ*B in rats of different treatment and expressions of the downstream cytokines IL-6 and IL-1*β* were assessed by WB methods. We found Tan IIA lead to decline in the expression of p-p65-NF-*κ*B, IL-6, and IL-1*β* of the tumor samples in comparison with the controls (Figure 3, *p* < 0.01); meanwhile, intestinal dysbacteriosis condition can increase the phosphorylation of p65, IL-6, and IL-1*β* in Tan IIA-treated mice (Figure 3, *p* < 0.01).

## 4. Discussion

GC is deemed to be a leading cause of death worldwide [18, 19]. Although patients with GC have benefited from chemotherapy with the improved overall survival, current chemotherapeutic agents have serious side effects in patients. Therefore, the discovery and development of the specific molecular targets necessitate modulation in anticancer therapy.

The role of the gut microbiome in a variety of cancers have been documented in many former studies, and now, intestinal dysbacteriosis has been identified as an important reason in the development of cancers [20, 21]. In the present work, we discovered that the intestinal microbiome significantly altered in the GC tumor mice in comparison with the control mice, while the beneficial microorganism *Lactobacillus* as well as *Bacteroides* decreased, and the harmful microorganism *Escherichia* as well as *Candidatus* increased. These results were consistent with previous observation [22], suggesting that intestinal dysbacteriosis may contribute to the pathogenesis of GC.

The antitumor influences of Tan IIA have been discussed in many previous studies. For example, Tan IIA inhibits ovarian cancer growth by suppressing malignant properties [23]. Tan IIA reduces colorectal cancer cell viability by activating JNK-Mff signaling pathways [24]. More importantly, Tan IIA has been also reported to hinder GC progression [25] but reports on the potential of Tan IIA in the gut microbiome of GC is rare. In this work, we first elucidated the potential Tan IIA in the intestinal microbiome. It was discovered that Tan IIA elevated the abundant of the useful microorganism whereas lessened the abundance of baleful microorganism in GC mice, and interestingly, when intestinal dysbacteriosis condition was created in Tan IIA-treated mice, the antitumor effects of Tan IIA has been partially blocked. Taken together, the above data mirrored that Tan IIA could exert its anti-GC influences in part via modulating the intestinal microbiome.

Intestinal dysbacteriosis was famous to trigger chronic inflammatory condition and consequentially contribute to the tumorigenesis. NF-*κ*B was known as a complex of proteins that take part in the progression of immune responses [26, 27]. As reported before, the NF-*κ*B pathway is involved in the regulation of intestinal microbiome in many diseases, such as colitis [28] and colorectal cancer [29], and its downstream cytokine IL-6 and IL-1*β* are closely related to the gut microbiota of GC [30]. Consistent with the above studies, the current work found that Tan IIA weakened p65-NF-*κ*B phosphorylation along with the downstream cytokine IL-6 and IL-1*β* in GC tumors, and intestinal dysbacteriosis could partially block the anti-inflammatory influences of Tan IIA. These outcomes suggested that Tan IIA may influence the intestinal microbiome via modulation of the NF-*κ*B signaling.

There are several limitations in our study. First, the potential mechanism of Tan IIA on regulating the NF-*κ*B pathway was not further explored. In addition, the type of gut microbiota examined in our study was few. Therefore, more researches are needed to further explore the clinical value of Tan IIA in GC.

## 5. Conclusion

In a word, we firstly reported that Tan IIA could hinder GC tumor growth via modulating the intestinal microbiome, maybe through inactivating the NF-*κ*B signaling. Our work may provide basis for the using of Tan IIA as a useful medication for GC therapy.

## Figures and Tables

**Figure 1:** Tan IIA influences GC tumor growth. (a) Images of the tumors in different groups. (b) Tumor volume measurement. (c) Tumor weight measurement. ^∗^*p* < 0.05, ^∗∗^*p* < 0.01.

**Figure 2:** Intestinal dysbacteriosis condition partially blocked Tan IIA-induced antitumor effects. (a) Images of the tumors in different groups. (b) Tumor volume measurement. (c) Tumor weight measurement. ^∗^*p* < 0.05, ^∗∗^*p* < 0.01.

**Figure 3:** Intestinal dysbacteriosis abrogated Tan IIA-stimulated decrease in the NF-*κ*B signaling in xenograft tumor mice. (a) Expression of NF-*κ*B and p-NF-*κ*B in different groups. (b) IL-6 level assessment. (c) IL-1*β* level assessment. ^∗∗^*p* < 0.01.

**Table 1:** Comparison of the abidance of intestinal microbiome between the GC tumor mice and the control mice.

	Control	Tumor	*p* value
*Lactobacillus*	33.24 ± 2.86	13.51 ± 1.35	*p* < 0.01
*Bacteroides*	32.05 ± 2.33	19.25 ± 1.86	*p* < 0.01
*Escherichia*	0.01 ± 0.01	2.21 ± 0.13	*p* < 0.001
*Candidatus*	2.09 ± 0.24	8.25 ± 0.32	*p* < 0.001

**Table 2:** Comparison of the abidance of intestinal microbiome between the GC tumor mice with or without Tan IIA treatment.

	Tumor	Tan IIA low	Tan IIA high
*Lactobacillus*	11.92 ± 1.43	19.02 ± 2.15	26.89 ± 3.04^∗∗^
*Bacteroides*	18.92 ± 1.75	23.49 ± 1.28^∗^	28.71 ± 2.85^∗^
*Escherichia*	2.33 ± 0.41	1.53 ± 0.21	0.29 ± 0.01^∗∗^
*Candidatus*	7.95 ± 0.72	4.84 ± 0.53^∗^	3.22 ± 0.71^∗∗^

^∗^ *p* < 0.05, ^∗∗^*p* < 0.01.

## Data Availability

Data included in the present study are available from the corresponding author under reasonable requests.

## Abbreviations

GC: Gastric cancer
Tan IIA: Tanshinone IIA
EMT: Epithelial-mesenchymal transition
FBS: Fetal bovine serum
SPF: Specific pathogen-free
PBS: Phosphate buffer saline
RIPA: Radio immunoprecipitation assay
ELISA: Enzyme-linked immunosorbent assay
IL-6: Interleukin-6
IL-1*β*: Interleukin-1*β*
NF-*κ*B: Nuclear factor kappa-B.
